The article "Single-Cell RNA Sequencing in Human Retinal Degeneration Reveals Distinct Glial Cell Populations" was published in 2020. Journal: Cells.

# Single-Cell RNA Sequencing in Human Retinal Degeneration Reveals Distinct Glial Cell Populations

**DOI:** 10.3390/cells9020438

**Published:** 2020-02-13

**Authors:** Andrew P. Voigt, Elaine Binkley, Miles J. Flamme-Wiese, Shemin Zeng, Adam P. DeLuca, Todd E. Scheetz, Budd A. Tucker, Robert F. Mullins, Edwin M. Stone

**Affiliations:** 1 Department of Ophthalmology and Visual Sciences, The University of Iowa Carver College of Medicine, Iowa City, IA 52242, USA; 2 Institute for Vision Research, The University of Iowa, Iowa City, IA 52242, USA

**Keywords:** autoimmune retinopathy, retinal degeneration, Müller cell, single-cell

## Abstract

Degenerative diseases affecting retinal photoreceptor cells have numerous etiologies and clinical presentations. We clinically and molecularly studied the retina of a 70-year-old patient with retinal degeneration attributed to autoimmune retinopathy. The patient was followed for 19 years for progressive peripheral visual field loss and pigmentary changes. Single-cell RNA sequencing was performed on foveal and peripheral retina from this patient and four control patients, and cell-specific gene expression differences were identified between healthy and degenerating retina. Distinct populations of glial cells, including astrocytes and Müller cells, were identified in the tissue from the retinal degeneration patient. The glial cell populations demonstrated an expression profile consistent with reactive gliosis. This report provides evidence that glial cells have a distinct transcriptome in the setting of human retinal degeneration and represents a complementary clinical and molecular investigation of a case of progressive retinal disease.

## 1. Introduction

Photoreceptor cells are highly specialized, terminally differentiated neurons that detect photons of light and transmit this information to bipolar cells in the retina. Unfortunately, their exacting structural and metabolic requirements make them very susceptible to a large number of acquired and genetic sources of injury, leading to irreversible vision loss [1]. Degenerative diseases affecting photoreceptor cells have multiple etiologies. For example, genetic variants in over 100 genes have been shown to cause heritable photoreceptor degeneration [2]. However, photoreceptor degeneration can also be immune mediated, as in the case of autoimmune retinopathy (AIR), where circulating retinal autoantibodies lead to inflammation and downstream photoreceptor destruction [3]. Photoreceptor loss can also occur secondary to damage or dysfunction of adjacent cells and extracellular structures; for example, diseases affecting the retinal pigment epithelium (RPE), Bruch’s membrane, or choroid can lead to increased oxidative stress and decreased metabolic support to the outer retina [4].

One approach for studying retinal degeneration is to characterize transcriptomic changes within diseased retina using microarrays or, more recently, next-generation sequencing of cDNA libraries (RNA sequencing, or RNA-Seq). Conventional gene expression studies with RNA-Seq have analyzed pools of retinal RNA from numerous cell types [5,6]. However, the high degree of cellular complexity and diversity in the human retina can prevent detection of even large gene expression changes that are restricted to specific classes of cells that are relatively unrepresented in the pool [7]. This concern has been largely obviated by the development of single-cell RNA sequencing, which has recently been employed to characterize the transcriptome of individual retinal cell populations. The neural retina is well suited for dissociation into single-cells, and protocols for recovery of viable, singlet cells are well established [8,9]. Such protocols facilitated the exploration of the murine retina transcriptome in the first report of Drop-Seq single-cell RNA sequencing [10]. Since this initial investigation, several additional studies have described the transcriptome of murine retina [10,11,12] and more recently, human retina [13,14,15] at the single-cell level.

In this report, we describe the clinical course of a 70-year-old patient with progressive photoreceptor degeneration attributed to AIR. We perform single-cell RNA sequencing on paired foveal and peripheral retinal samples from this patient and four unaffected control patients to investigate how different populations of retinal cells respond to photoreceptor degeneration. A total of 23,429 cells were recovered in this experiment, including 7189 cells from the AIR patient. This study provides insight into the responses of the retina to a blinding inflammatory condition at the cellular and transcriptional levels.

## 2. Materials and Methods

Human Donor Eyes: Eyes from the human donors utilized for this study were acquired from the Iowa Lions Eye Bank in accordance with the Declaration of Helsinki and following full consent of the donors’ next of kin. The Institutional Review Board at the University of Iowa has judged that experiments performed on the donated eyes of deceased individuals does not fall under human subjects rules. All of the experiments in present paper were on the eyes of deceased individuals donated to science by the donors’ next of kin. The work we performed in this paper was not human subjects research. Donor information is presented in Table 1. All tissue was received in the laboratory within 7 h post-mortem and processed immediately. A 2 mm foveal centered punch and an 8 mm peripheral retinal punch from the inferotemporal region centered on the equator were acquired with a disposable trephine from each donor. For the AIR donor, the OS was used for single-cell RNA sequencing and the OD was preserved in freshly generated 4% paraformaldehyde in phosphatidylcholine buffer solution. Frozen sections from the macula and peripheral retina were prepared as described previously [16]. Sections were stained with hematoxylin-eosin stain.

Dissociation for single-cell analysis: The overlying retinal tissue was peeled off of the retinal pigment epithelium and choroid. Retinal tissue was subsequently dissociated in 20 units/mL of papain with 0.005% DNase I (Worthington Biochemical Corporation, Lakewood NJ) for 1.25 h on a shaker at 37 °C. Dissociated cell suspensions were frozen in DMSO-based Recovery Cell Culture Freezing Media (Life Technologies Corporation, Grand Island NY) in a Cryo-Safe cooler (CryoSafe, Summerville SC) to cool at 1 °C/min at −80 °C for 3–8 h before storage in liquid nitrogen.

Sample Preparation: Cryopreserved retinal samples were rapidly thawed and resuspended in phosphatidylcholine buffer solution with 0.04% non-acetylated bovine serum albumin (New England Biolabs, Ipswich, MA, USA) at a concentration of 1000 cells/μL. Viability analysis was performed with the Annexin V/Dead Cell Apoptosis Kit (Life Technologies Corporation, Eugene, OR, USA), with viability >90% using the Countess II FL Automated Cell Counter (ThermoFisher Scientific, Waltham, MA, USA). Next, single cells were captured and barcoded using the Chromium system v3.0 chemistry kit (10X Genomics, Pleasanton, CA, USA). Barcoded libraries were pooled before sequencing on the HiSeq 4000 platform (Illumina, San Diego, CA, USA), generating 150 base pair paired-end reads.

Immunohistochemistry: Immunohistochemical experiments were performed on frozen tissue sections from donor eyes fixed in 4% paraformaldehyde. Sections were blocked with 1 mg/mL of bovine serum albumin before one-hour incubation with anti-ANXA1 (1:1.7, Developmental Studies Hybridoma Bank, Iowa City, IA) or Blue Cone Opsin (1:200, Millipore, AB5407), Red/Green Cone Opsin (1:200, Millipore, AB5405), and RetP1 (1:1000, Thermo Scientific). Sections were subsequently washed and incubated with Alexa-546-conjugated anti-mouse IgG (1:200, Invitrogen) or Alexa-488-conjugated anti-mouse IgG (1:200, Invitrogen) and Alexa-546-conjugated anti-rabbit IgG (1:200, Invitrogen). Each secondary antibody was supplemented with 100 μg/mL diamidino-phenyl-indole (DAPI, Sigma). Sections were incubated for 30 min before washing and cover slipping. Negative controls were included by omitting each primary antibody. Sections were photographed with an epifluorescent microscope (Olympus BX41) equipped with a digital camera (SPOT-RT; Diagnostic Instruments).

Computational Analysis: In addition to the two new donors sequenced for this study, we recently reported single-cell RNA sequencing on paired foveal (2 mm) and peripheral neural retina isolated from three human donors [13] with identical sample processing. FASTQ files from the previous experiment (n = 3 paired samples, donors 1-3; GSE130636) and the current experiment (n = 2 paired samples, donors 4–5) were utilized for downstream analysis. Briefly, FASTQ files were generated from basecalls with the bcl2fastq software (Illumina, San Diego, CA, USA) by the University of Iowa Institute of Human Genetics. Next, FASTQ files were mapped to the hg19 genome with CellRanger (v3.0.1) [17]. Cells with unique gene counts fewer than 200 were filtered, and cells with greater than 7000 unique genes per cell were removed to eliminate potential doublets. Libraries were aggregated to the same effective sequencing depth, and log-normalization of aggregated reads was performed with Seurat (v2.3.4) using a scale factor of 10,000 [18]. All raw and processed data have been deposited in NCBI’s Gene Expression Omnibus (GSE142449).

## 3. Results

### 3.1. Patient Description

The patient initially presented to the neuro-ophthalmology service at the age of 51 for evaluation of decreased peripheral visual fields and photopsias in both eyes. He had no family history of inherited retinal degeneration. At presentation, his visual acuity was 20/20 in each eye, but he was found to have peripheral visual field loss. Ophthalmoscopic examination early in his disease course showed granular juxtapapillary pigmentary changes and mild vascular attenuation in both eyes. Electroretinogaphy (ERG) at presentation was consistent with widespread retinal dysfunction affecting both rods and cones. He experienced relatively rapid progression of his visual field loss and was seen by the inherited retinal degeneration service with concern for retinitis pigmentosa versus autoimmune retinopathy (AIR). Cancer-associated retinopathy was also considered, but his workup for malignancy was negative and his ERG was felt to be inconsistent with a paraneoplastic process at that time.

He ultimately developed peripheral bone-spicule-like pigmentary changes in both eyes (Figure 1A,B, 7 years after initial presentation) and progressive visual field constriction (Figure 1C,D, 8 years after initial presentation). Molecular evaluation for an inherited retinal degeneration, including whole exome sequencing, was performed but failed to identify a genetic etiology for his condition (for methods see [2]). He developed colon cancer several years after presentation, but this was thought to be unrelated to his ocular disease. He was given a presumed diagnosis of autoimmune retinopathy and ultimately required treatment for cystoid macular edema with intravitreal steroids.

At the time of his last follow up with the retina service at the age of 69, his visual acuity was 20/40 + 1 in the right eye and 20/100 in the left eye with stable peripheral pigmentary changes in both eyes, and no cystoid macular edema. At age 70, the patient expired and donated his eyes for ophthalmic research. Evaluation of the patient’s serum with Western blotting revealed the presence of antibodies that reacted with a 23 kilodalton protein in human retina.

### 3.2. Histological Findings

Sections from an eye with normal ocular history (Figure 2A), from the macula of the AIR donor (in the OD, the eye with better visual acuity) (Figure 2B), and from the periphery of the AIR donor (Figure 2C,D) were acquired. The macula of the AIR donor showed a loss of rod photoreceptors with only a single layer of attenuated cone cells remaining. In spite of the photoreceptor cell loss, the RPE was confluent and the inner retina appeared intact, with discrete inner nuclear layers and ganglion cell layers. In the periphery, the AIR donor showed complete loss of inner and outer segments and of the outer nuclear layer (Figure 2C). Considerable pigment migration into the inner retina was also observed in the periphery of the AIR donor (Figure 2D).

Cone and rod photoreceptor cells were also visualized with fluorescent immunohistochemistry (IHC). Within the macula of a donor with normal ocular history, abundant cone opsin and rhodopsin labeling was observed (Figure 2E). In contrast, the AIR donor demonstrates complete loss of the rod specific opsin rhodopsin as well as extreme attenuation of cone photoreceptors (Figure 2F).

### 3.3. Single-Cell Gene Profiling of Diseased Cell Populations

Paired foveal and peripheral retinal punches were acquired from each of the five donors. While the four control donors had grossly normal retinas upon examination in the laboratory (Figure 3A), the donor with AIR had abundant peripheral pigmentation with a mostly unaffected macula (Figure 3B). After gentle dissociation, single-cell RNA sequencing was performed on each foveal and peripheral sample, and a total of 23,429 cells were recovered after filtering (Figure 3C). A total of 23 clusters were identified, and expression profiles were used to assign each cluster to its corresponding retinal cell type (Figure 3D). All major populations of retinal neurons, as well as supporting retinal endothelial cells, pericytes, glial cells, and microglia, were identified.

Next, the distribution of recovered cell types was compared between the AIR donor and the four control donors (Table S1). As the cellular composition of the retina varies between the fovea and periphery, comparisons were stratified by region. Within the fovea, cone photoreceptor cells are more abundant than rod photoreceptor cells, and cone photoreceptor cells synapse one-to-one with bipolar cells and upstream retinal ganglion cells (Figure 4A). The fovea centralis comprises the central 0.65-0.70 mm of the retina, consisting exclusively of cone photoreceptor cells and excluding vascular elements [19]. Our use of 2 mm foveal centered punches completely captures the fovea centralis but also includes some central rod photoreceptors and retinal endothelial cells. In the four control donors, all major populations of inner retinal neurons were recovered from the fovea (Figure 4B). No RPE cells were detected, suggesting that the foveal retinal punch was well separated from the underlying RPE and choroid. Unlike the control donors, no rod photoreceptor cells were detected in the foveal punch from the donor with AIR. However, a similar proportion of foveal cone photoreceptor cells were recovered in the AIR donor and the control donors. In addition, the AIR donor demonstrated a moderate increase in the proportion of recovered foveal bipolar and Müller cells.

In the periphery, rod photoreceptor cells were predominant, and peripheral bipolar cells receive input from multiple rod photoreceptor cells (Figure 4D). In the four control donors, peripheral rod photoreceptor cells were much more abundant than cone photoreceptor cells, and relatively few microglia or astrocytes were detected (Figure 4E). In contrast, only a single rod photoreceptor cell was recovered from the periphery of the AIR donor while microglia and astrocyte cells were recovered in much higher frequency. In addition, a small proportion of RPE cells were recovered from the periphery of the AIR donor, consistent with the histological observation of peripheral RPE migration into the retina (Figure 2D).

Next, the transcriptomic consequences of photoreceptor degeneration in the AIR donor were investigated. For each cell type, gene expression was compared between cells originating from the AIR donor and the control donors, and the proportion of significantly differentially expressed genes (adjusted *p*-value < 0.05) that exhibited an absolute log fold-change in expression greater than 0.5 was calculated. As gene expression within a single cell type can vary between the fovea and the periphery [13], this analysis was again stratified by region. Within the fovea, Müller cells and horizontal cells demonstrated modest expression differences, with a total of 1.1% and 1.2% of assayed genes significantly enriched in the AIR Müller cell and horizontal cell populations, respectively (Figure 4C). A greater proportion of differentially expressed genes between the AIR and control donors were identified in the periphery (Figure 4F). Müller and astrocyte glial cells both demonstrated a modest proportion of genes significantly enriched in the periphery of the AIR donor (1.3% and 2.1%, respectively), as did microglia and horizontal cells (2.2% and 2.6%, respectively). Differential expression results for each comparison are shown in detail in Table S2.

While most clusters contained cells from each of the five donors, Clusters 4–6 were comprised predominantly of cells from the periphery of the AIR patient (each cluster possessing >85% of cells from the AIR donor) (Figure 5A). Therefore, gene expression patterns from these clusters were further investigated. Cluster 4 was classified as astrocytes (Figure 5C,D). Cells in this cluster demonstrated high expression of the glial fibrillary acid protein (GFAP), which is widely expressed in astrocytes responding to neuronal injury [20], and the astrocyte-specific inflammatory cytokine IFITM3 [21]. A total of 624 cells were recovered in Cluster 4 and 551 of them (88%) originated from the periphery of the AIR donor. Differential expression analysis was performed to investigate if astrocytes from the AIR donor demonstrated a reactive gene expression profile (Figure S1). Astrocytes from the AIR donor were enriched for SOCS3 [22], SLPI [23], and CH25H [24], genes that have all been previously found to be expressed in astrocytes responding to CNS injury. In addition, reactive glial cells are involved in inflammatory responses, and have been shown to increase the production of pro-inflammatory chemokines [25]. The chemokine CXCL2 was highly enriched (logFC = 1.47) in peripheral astrocytes from the AIR donor.

Cluster 5, with 98% of cells originating from the periphery of the AIR donor, was interpreted as Müller glial cells. Cells in this cluster highly expressed the Müller cell genes RLBP1 and CRALBP1 (Figure 5E). Six additional clusters of Müller glia were identified, which largely separated Müller cells of peripheral (Clusters 6–10) and foveal (Clusters 11–2) origin (Figure 5A). As previously shown in monkey [26] and human [13] retina, foveal and peripheral Müller cells have distinct gene expression profiles (Figure 5G). Interestingly, foveal Müller cells from the AIR donor clustered with foveal Müller cells from the other four donors, and differential expression analysis yielded relatively few expression differences (log fold-change greater than 1.25) (Figure 5H). NFKBAI, which has been previously associated with glial cell degeneration, [27] was the most upregulated gene in the AIR donor’s foveal Müller cells.

In contrast, the majority of peripheral Müller cells from the AIR donor formed their own cluster (Cluster 5). Differential expression revealed numerous expression differences between peripheral Müller cells from the AIR donor versus peripheral Müller cells from other donors (Figure 5I). Among the first hallmarks of reactive gliosis is the increased expression of intermediate filament proteins [28]. The intermediate filament gene GFAP (logFC = 2.54) was the most enriched gene in Müller cells from the AIR donor, which was also observed to be more abundant in the AIR donor at the protein level (Figure S2). In addition, peripheral Müller cells from the AIR donor were enriched for ANXA1 and ANXA2, which have been shown to be upregulated in reactive glial populations in the brain [29]. Immunofluorescent IHC also demonstrates increased ANXA1 labeling in cells of the AIR donor (Figure 5B), which co-localizes with GFAP expression (Figure S3).

Cluster 6, with 99% of cells originating from the periphery of the AIR donor, was interpreted as retinal pigment epithelium (RPE) cells (Figure 5F). Cells in this cluster demonstrated high expression of SERPINF1 (the gene encoding PEDF) and RLBP1 (the gene encoding cellular retinaldehyde binding protein). Although retinal samples were dissected away from the underlying RPE and choroid, the recovery of RPE cells suggests that either some RPE cells migrated into the inner retina or remained adhered to the outer retina after dissection, consistent with both the clinical observation of bone spicule like pigmentation in the patient’s neurosensory retina (Figure 1A–B) and the morphological finding of pigment migration into the inner retina (Figure 2D).

## 4. Discussion

Autoimmune retinopathy (AIR) is a blinding, immune-mediated inflammatory condition in which anti-retinal antibodies result in retinal cell destruction. In most cases, photoreceptor cells are the primarily targeted cell type, although antibodies against bipolar cells have also been reported [30]. The clinical presentation of the patient in this report follows the classical trajectory of sudden, bilateral loss of peripheral vision, consistent with rod photoreceptor cell dysfunction [31]. The etiology of AIR is broadly subdivided into paraneoplastic and non-paraneoplastic disease. Identifying anti-retinal antibodies can support a diagnosis of AIR, however unaffected individuals may also have circulating anti-retinal antibodies, limiting the specificity of this diagnostic assay [32,33].

Consistent with the clinical history of peripheral visual deterioration, histological examination of the AIR patient revealed a profound loss of both cone and rod photoreceptor cells and destruction of the inner and outer photoreceptor segments in the periphery (Figure 2C). However, in the macula, rare attenuated cone photoreceptor cells were still present (Figure 2F). Single-cell RNA sequencing supported these clinical and histological findings. Only a single rod photoreceptor cell was recovered from the periphery of the AIR donor while numerous foveal cones were recovered. In addition, single-cell RNA sequencing identified the presence of RPE cells in the periphery of the AIR donor, as was observed on histological examination (Figure 2D). Gene expression comparisons between the AIR donor and the four control donors were remarkably similar for most cell types. However, peripheral astrocytes and Müller glial cells were more abundant and demonstrated unique expression signatures in the AIR patient. Collectively, these expression data corroborate the clinical and histologic findings and provide evidence that single-cell RNA sequencing can be a complementary tool for investigating the molecular features of a human retinal disease.

The retina contains two major classes of glial cells: Müller cells and astrocytes. Müller cells are elongated cells that extend from the external limiting membrane (apical end) to the internal limiting membrane (basal feet). Müller cells provide metabolic and structural support to retinal neurons, ensheathing neural somas and comprising an important part of the blood retina barrier. Astrocytes also metabolically support the retina, however astrocytes do not originate from the embryonic retinal neuroepithelium but rather enter the retina by migrating along the developing optic nerve [34]. As opposed to Müller cells, astrocytes are star-shaped cells with radiating processes located in the nerve fiber and ganglion cell layers. Both astrocytes and Müller glial cells are capable of responding to retinal injury and exerting neuroprotective effects on the retina in a process known as reactive gliosis [35]. In this wound response process, glial cells proliferate and undergo changes in gene expression for improved neuronal protection and repair [36,37].

In the donor with AIR, the transcriptional response of the glial cells can likely be attributed to their interactions with degenerating retina. Within the fovea, where the retina clinically and histologically was most intact, Müller cells from the AIR donor were transcriptionally similar to foveal Müller cells from the control patients. Yet in the peripheral retina, where the AIR donor experienced progressive visual field loss and a complete loss of the outer nuclear layer, peripheral Müller cells segregated into a distinct cluster and demonstrated a reactive gliotic phenotype (Figure 5I). Likewise, many astrocytes were recovered from the periphery of the AIR donor that expressed genes implicated in reactive gliosis (Figure S1). Reactive astrogliosis is marked by astrocyte proliferation and migration, which may have led to an increased number of peripherally localized astrocytes available for recovery in the AIR donor, consistent with recent single-cell RNA sequencing studies characterizing microglial proliferation in response to retinal damage in mice [38]. Collectively, the gliotic injury response induced by Müller cells and astrocytes has many neuroprotective benefits, yet chronic gliotic activation can further injure retinal neurons and disrupt the blood–retinal barrier, leading to worsening vision [39,40]. In the setting of chronic retinal injury, interventions that modulate gliotic activation may optimize preservation of remaining retinal function [41].

While glial cells from the AIR donor demonstrated reactive transcriptional changes, most inner retinal cell populations from this donor had remarkably similar gene expression profiles to the control donors (Figure 4C,F). Likewise, histological examination revealed preserved inner retinal morphology with discrete inner nuclear and ganglion cell layers (Figure 2B,C). Collectively, these findings suggest that even in the setting of photoreceptor cell degeneration, the inner retinal wiring remains largely undamaged. The presence of morphologically and transcriptomically normal inner retinal cells is promising for prospective photoreceptor degeneration treatments, including autologous retinal cellular replacement strategies [42].

There are several limitations to this study. First, AIR is a rare retinal disease, preventing us from including multiple patients with this condition in this investigation. As a result, gene expression differences between the AIR donor and the four control donors are valuable for hypothesis generation but should be interpreted with caution. Second, while all samples had identical sample processing, certain cell types might have a selective advantage in cellular recovery for single-cell RNA sequencing. Recovered proportions of cells at the single-cell level (Figure 4B,E) should not be interpreted as the true cellularity of the retina.

This study provides a complementary investigation of the clinical and molecular response of the retina in AIR. Clinical, histologic, and transcriptomic evidence identify the loss of cone and rod photoreceptor cells with relative preservation of inner retinal cell types. The gliotic transcriptional profile of astrocyte and Müller glial populations observed in this case provides some new insight into the retina’s response to photoreceptor degeneration.

## Figures and Tables

**Figure 1:** Clinical findings in a patient with retinal degeneration. (**A**,**B**): Montage color fundus photographs of the right (**A**) and left (**B**) eyes. There was granular, retinal pigment epithelial atrophy in the mid-periphery of both eyes, in addition to peripheral bone-spicule-like pigmentary changes and pigment clumps in both eyes. Arteriolar attenuation was notable in both eyes. (**C**,**D**): Goldman visual fields of the right (**C**) and left (**D**) eyes. There was severe constriction of the peripheral visual field in both eyes.

**Figure 2:** Histological and immunohistochemical investigation of the autoimmune retinopathy (AIR) and control donors. (**A**–**D**). Hematoxylin and eosin staining of the AIR and control donors. Sections from the periphery of a control donor (donor 2) (**A**), the macula (OD) of the AIR donor (**B**), and the periphery of the AIR donor (**C**,**D**). The AIR macula demonstrates intact ganglion cell and inner nuclear layers with attenuated cone photoreceptor outer segments. In contrast, in the periphery of the AIR donor complete loss of the outer nuclear layer (**C**) and retinal pigment epithelium (RPE) pigment migration into the inner retina (**D**) is observed (*). (**E**,**F**): Cone opsins (blue cone opsin and red/green cone opsins) are labeled in red while RetP1 is labeled in green. (**E**): A macula from a donor with normal ocular history demonstrates abundant labeling of cone opsins and rhodopsin. Of note, the RPE below the photoreceptors is out of frame. (**F**) The macula from the AIR donor demonstrates a complete lack of rod photoreceptors with rare, extremely attenuated cone photoreceptors (arrows). Autofluorescent lipofuscin from the RPE appears below the photoreceptor cells. Scalebar (100 microns) for all subpanels is provided in (**E**).

**Figure 3:** Single-cell RNA sequencing of the AIR donor. (**A**,**B**): Five human donor eyes were used for this study. A gross image of a control eye (donor 4) (**A**) and the AIR eye (donor 5) (**B**) are included. From each eye, a 2 mm foveal centered punch (red) and an 8 mm peripheral punch isolated from the inferotemporal region (blue) were acquired and gently dissociated. Scalebar (**A**) is 5 mm. (**C**): Single-cell RNA sequencing of retinal cells from the AIR donor and four control patients. A total of 23,429 cells were recovered after filtering. Unsupervised clustering of cells resulted in 23 clusters, which are visualized with uniform manifold approximation and projection (UMAP) dimensionality reduction, where each point represents the multidimensional transcriptome of a single-cell and each cluster of cells is depicted in a different color. (**D**): Violin plots depict the expression of cell-type specific genes across the 23 identified clusters. Per = peripheral retina. AIR = autoimmune retinopathy. RPE = retinal pigment epithelium. RGC = retinal ganglion cell.

**Figure 4:** Library composition of recovered cells. (**A**): In the fovea, cone photoreceptor cells synapse with one bipolar cell, which synapse with one retinal ganglion cell. (**B**): The proportion of each cell type recovered from the fovea of the four control donors and the autoimmune retinopathy donor. No foveal rods were recovered from the AIR donor. (**C**): In order to visualize the degree of gene expression differences within each population of cells between the AIR and control donors, differential expression analysis was performed. In each cell type, the number of differentially expressed genes that were enriched in the AIR donor and the control donors were enumerated and divided by the total number of expressed genes (in at least 10% of cells). For example, 1.09% of foveal Müller cell genes were significantly enriched in the AIR donor (dark grey), while 0.57% of foveal Müller cell genes were significantly enriched in the control donors (light grey). (**D**): In the periphery, multiple rod photoreceptor cells synapse with a single bipolar cell. (**E**): The proportion of each cell type recovered from the periphery of the four control donors and the periphery of the AIR donor. (**F**): As in (**C**), the proportion of differentially expressed genes between the AIR and control donors was performed in each cell type. More genes were differentially expressed in the periphery compared to the fovea (**C**). As no RPE cells originated from control donors, differential expression could not be performed in the periphery for this cell type.

**Figure 5:** Exploration of autoimmune retinopathy dominant clusters. (**A**): The library composition of each cluster is displayed, with cells originating from the control foveas represented in shades of blue while cells originating from the control peripheries are in shades of green. Cells originating from the AIR donor are colored light red (fovea) or dark red (periphery). Three clusters (Cluster 4–6) consist predominantly of cells from the periphery of the AIR donor. (**B**): Immunofluorescent labeling of ANXA1 in the retina of a control donor (left) and the AIR donor (right). The AIR donor demonstrates increased ANXA1-labeling of the inner retina. Scale bar = 100 microns. (**C**): Violin plots of SOCS3, GFAP, RLBP1, and SERPINF1 expression are used to classify the cell types of clusters 4–6. (**D**): Cluster 4 specifically expressed SOCS3, which is enriched in reactive astrocytes. (**E**): Cluster 5 and Clusters 7-12 express the Müller cell specific gene RLBP1. (**F**): Cluster 6 expresses the RPE-specific gene SERPINF1. (**G**): Healthy foveal and peripheral Müller cells have distinct gene expression profiles. The variable delta percent along the x-axis represents the proportion of foveal Müller cells that express the gene of interest minus the proportion of peripheral Müller cells that express that gene. (**H**): Foveal Müller cells originating from the control donors have similar gene expression profiles to foveal Müller cells originating from the AIR donor. (**I**): In contrast, peripheral Müller cells from control versus the AIR donor demonstrated more transcriptomic differences. Genes with a log fold-change greater than 1.0 and a delta percent greater than 0.35 are labeled in (**G–I**).

**Table 1:** Sample information from the donor eyes utilized in this study. Note that donor eyes 1–3 serve as controls for the current study and have been previously published [13].

Donor	Age	Sex	Time Postmortem	Eye	Cause of Death	Ophthalmologic History
Donor 1	89	Male	5:21	OD	Cancer	Early stage glaucoma documented; histologically normal
Donor 2	54	Male	5:29	OD	Cardiac arrest	No records received; histologically normal
Donor 3	82	Female	4:18	OD	Cardiopulmonary arrest	No ophthalmic records; histologically normal
Donor 4	76	Male	5:14	OS	Respiratory failure/cancer	posterior vitreous detachment OU, nuclear sclerosis OU; histologically normal
Donor 5	70	Male	6:36	OS	Chronic obstructive pulmonary disease	AIR, see results 3.1

## Supplementary Materials

The following are available online at https://www.mdpi.com/2073-4409/9/2/438/s1, Figure S1: AIR astrocytes demonstrate a reactive gene expression profile. Figure S2: Increased GFAP in the AIR donor versus a healthy control donor. Figure S3 ANXA1 and GFAP co-localization in the AIR donor. Table S1: Library Composition, Table S2: Differential expression between the AIR donor versus four control donors.
